The article "Bactrim-Induced Hepatotoxicity" was published in 2024. Journal: Cureus.

# Bactrim-Induced Hepatotoxicity

**DOI:** 10.7759/cureus.74053

**Published:** 2024-11-19

**Authors:** Henry Onyirimba, Ava L Boudi, Max Boudi, Connie S Chan, F Brian Boudi

**Affiliations:** 1 Medicine, Banner Health, Phoenix, USA; 2 Science, Arizona State University, Phoenix, USA; 3 Education, Arizona State University, Phoenix, USA; 4 Internal Medicine, University of Arizona College of Medicine, Phoenix, USA; 5 Cardiology, University of Arizona College of Medicine, Phoenix, USA

**Keywords:** allergic reaction, cholestatic jaundice, drug-related side effects and adverse reactions, hepatic toxicity, treatment-related toxicity

## Abstract

Sulfamethoxazole/trimethoprim (SMX/TMP) is a commonly used antimicrobial agent for treating common bacterial infections such as urinary tract infection (UTI), combined with doxycycline for community-acquired methicillin-resistant* Staphylococcus aureus *(MRSA), and invaluable in *Pneumocystis jirovecii* pneumonia (PJP), previously classified as *Pneumocystis carinii*. Of its known adverse reactions, hepatotoxicity rarely comes to mind, but indeed, it is a recognized but very rare adverse reaction that may lead to liver failure in adults and even rarer in children. We present a case of hepatotoxicity in a 43-year-old male patient on no prior medication who developed jaundice and highly elevated liver enzymes one week after the administration of Bactrim for the treatment of UTI in association with prostatism, symptoms of decreased urinary force due to obstruction of flow through the prostate gland. He made a good recovery over several weeks with discontinuation of the medication and supportive care.

## Introduction

Sulfamethoxazole/trimethoprim (SMX/TMP), also known by brand names such as Bactrim and Septra, is a sulfonamide antibiotic used extensively in treating various bacterial infections. This combination antibiotic includes sulfamethoxazole, a sulfonamide that inhibits bacterial synthesis of dihydrofolic acid, and trimethoprim, which blocks the subsequent reduction to tetrahydrofolic acid, both of which are critical for bacterial DNA and protein synthesis. SMX/TMP achieves a bactericidal effect against many Gram-positive and Gram-negative bacteria by inhibiting these sequential steps in folate metabolism. Clinically, SMX/TMP is used for urinary tract infections (UTIs) and skin and soft tissue infections, including those caused by community-acquired methicillin-resistant *Staphylococcus aureus* (MRSA), and in prophylaxis against *Pneumocystis jirovecii* pneumonia (PJP) in patients with compromised immune systems. Despite its efficacy and frequent use, SMX/TMP is associated with several known side effects. These include hypersensitivity reactions, dermatologic effects, renal impairment, hematologic abnormalities, and electrolyte imbalances. Of these, hepatotoxicity is among the rarest but can be particularly concerning due to its potential severity. Hepatotoxicity with SMX/TMP is often defined as a twofold or greater elevation in liver enzymes or bilirubin from baseline values, and its severity can range from mild enzyme elevations to fulminant hepatic failure [1,2].

Drug-induced liver injury (DILI) remains a significant cause of acute liver failure in the United States, with antibiotics among the most common medications implicated in DILI cases [3]. Although hepatotoxicity from SMX/TMP is rare, it has been documented in multiple case reports and studies, underscoring the need for awareness among clinicians. Identifying SMX/TMP as a potential source of hepatotoxicity is crucial, as timely diagnosis and discontinuation of the offending agent can significantly improve patient outcomes. This report details a case of SMX/TMP-induced hepatotoxicity in an otherwise healthy adult male patient, discussing his clinical course, diagnostic findings, and the literature on mechanisms of SMX/TMP hepatotoxicity to aid in the recognition and management of this adverse reaction.

## Case presentation

A 45-year-old male patient with no known preexisting health conditions presented to the emergency department (ED) in September 2016 due to jaundice and markedly elevated liver enzymes. The patient had been in his usual state of health until three weeks before presentation when he was evaluated by his primary care physician (PCP) and diagnosed with benign prostatic hyperplasia (BPH) and a urinary tract infection. To address his symptoms of prostatism and suspected bacterial infection, the PCP referred him to a urologist, who subsequently prescribed a two-week course of SMX/TMP (one double-strength tablet containing 800 mg SMX and 160 mg TMP, twice daily) for the UTI and Flomax for BPH.

Within five days of initiating SMX/TMP therapy, the patient began experiencing generalized malaise, fatigue, and weakness, which he attributed to possible side effects of the antibiotic. Due to the worsening of his symptoms, he chose to discontinue SMX/TMP on day 7. However, his malaise persisted, and he soon noted yellow discoloration of his eyes. Concerned about these developments, he returned to his PCP, who ordered a comprehensive metabolic panel (CMP). The laboratory results were notable for an aspartate transferase (AST) of 2444 IU/L, alanine aminotransferase (ALT) of 3566 IU/L, alkaline phosphatase of 224 IU/L, and total bilirubin of 20.3 mg/dL, all suggestive of significant liver injury (Table 1). Given the severity of these abnormalities, he was advised to seek emergency care.

**Table 1:** Serial liver function testing with reference ranges (day 1-4) AST: aspartate aminotransferase, ALT: alanine aminotransferase, Alk-Phos: alkaline phosphatase, UDS: urine drug screen, ANA: antinuclear antibody, PCP: primary care physician

Parameter	Reference range	PCP	Day 1	Day 2	Day 3	Day 4
AST (U/L)	10-40	2444	2288	1988	1619	1463
ALT (U/L)	7-56	3566	3410	2806	2322	2158
Alk-Phos (U/L)	44-147	224	201	177	158	162
Total bilirubin (mg/dL)	0.1-1.2	13.4	20.3	18.6	18.1	17
UDS	Negative	Negative	Negative	-	-	-
Ethanol	Negative	-	Negative	-	-	-
Tylenol	Negative	-	Negative	-	-	-
ANA	Negative	-	Negative	-	-	-
Ceruloplasmin (mg/dL)	15-30	-	34	-	-	-

The patient denied any history of abdominal pain, pruritus, fever, recent travel, or known hepatitis exposure. His medical history was negative for alcohol use, recreational drugs, and contact with individuals diagnosed with hepatitis. Other than the recent use of SMX/TMP, his only medication was Flomax. Importantly, he had no history of over-the-counter or herbal medication use, minimizing the likelihood of other hepatotoxic agents. A hepatitis panel was negative for viral hepatitis A, B, and C, and imaging studies revealed no structural abnormalities in the liver, suggesting SMX/TMP as the most probable cause of his liver injury.

## Discussion

The patient's serial liver function tests showed markedly elevated AST, ALT, and total bilirubin levels, which are hallmarks of hepatocellular injury. The initial CMP results on day 1 revealed an AST level of 2444 IU/L and an ALT level of 3566 IU/L, far exceeding the normal range (AST: 10-40 U/L, ALT: 7-56 U/L). These elevated transaminase levels, combined with the patient's clinical symptoms of jaundice and malaise, align with known patterns of hepatocellular injury caused by SMX/TMP. The gradual decrease in these enzyme levels over subsequent days, as shown in Table 1, correlates with the discontinuation of SMX/TMP and the absence of other hepatotoxic agents, indicating a likely causative relationship.

Further analysis of the data underscores that while the patient's alkaline phosphatase level was only modestly elevated (224 U/L) (normal range: 44-147 U/L), the total bilirubin remained significantly high at 20.3 mg/dL. This pattern supports a primarily hepatocellular injury with some elements of cholestatic response, a mixed pattern commonly seen in SMX/TMP-induced hepatotoxicity. The sustained bilirubin elevation on day 4, despite decreasing transaminases, further corroborates this mixed injury pattern.

Although hepatotoxicity is a rare side effect of SMX/TMP, several case reports and studies document its potential for severe liver injury. The incidence of hepatotoxicity linked to SMX/TMP is estimated to be less than one in 10,000 exposures, with risk factors including immunosuppression and prolonged use [4,5]. An analysis of drug-induced liver injury cases in Denmark revealed that antibiotics, including SMX/TMP, accounted for 10% of DILI cases. However, SMX/TMP was responsible for a relatively small percentage [6]. This relatively low incidence often delays diagnosis, as clinicians may not initially consider SMX/TMP as a cause of liver dysfunction.

Notably, a 2014 Taiwanese study highlighted an increased incidence of liver function test abnormalities in HIV-positive patients on SMX/TMP for PCP, suggesting that immunocompromised patients may be more susceptible to SMX/TMP-related hepatotoxicity [7]. The study indicated that the immunocompromised state, combined with the complex metabolism of SMX/TMP, could contribute to a heightened risk of liver injury. Moreover, retrospective studies from the United States and Europe have shown that SMX/TMP hepatotoxicity can lead to varied presentations, ranging from mild liver enzyme elevations to fulminant hepatic failure necessitating liver transplantation [8,9].

Mechanisms of hepatic injury

SMX/TMP-induced hepatotoxicity is understood to occur through several complex mechanisms, each contributing to the diversity of its clinical presentations.

Hepatocellular Injury

SMX/TMP may cause direct hepatocyte damage by inhibiting mitochondrial function, leading to oxidative stress and reduced adenosine triphosphate (ATP) production. Mitochondrial toxicity disrupts oxidative phosphorylation, leading to hepatocyte death, inflammation, and elevated transaminases. This form of injury can be severe and is often associated with a rapid onset of symptoms [10-12].

Cholestatic Injury

In some cases, SMX/TMP metabolites interfere with bile excretion, leading to cholestatic jaundice. This pattern is typically characterized by elevated alkaline phosphatase and bilirubin levels, with modest transaminase increases. Cholestatic injury is less common with SMX/TMP but has been documented, particularly in older adults [13,14]. Cholestasis may result from an immune-mediated reaction that targets biliary epithelium, complicating presentation and management [15].

Mixed Pattern Injury

Patients may present with a combination of hepatocellular and cholestatic injury. This mixed pattern reflects both direct cytotoxic effects on hepatocytes and obstruction in bile flow, leading to simultaneous elevations in transaminases, alkaline phosphatase, and bilirubin [16].

Vanishing Bile Duct Syndrome (VBDS)

In rare cases, SMX/TMP-induced hepatotoxicity can result in VBDS, characterized by immune-mediated destruction of intrahepatic bile ducts. VBDS leads to progressive loss of bile ducts, cholestasis, and potentially irreversible liver damage. Documented cases of SMX/TMP-associated VBDS have required liver transplantation due to the progression of cholestatic liver disease [17,18]. This severe manifestation underscores the need for clinicians to recognize the potential for long-term complications with SMX/TMP hepatotoxicity.

Management and outcome

Upon discontinuing SMX/TMP, the patient's liver function tests were closely monitored, showing a gradual improvement over several weeks. Supportive care was provided, and liver enzymes and bilirubin levels trended toward baseline, consistent with previously documented recoveries from SMX/TMP hepatotoxicity where the injury was reversible [19]. Although no specific antidote exists for SMX/TMP-induced hepatotoxicity, early discontinuation of the drug is crucial for preventing further liver damage.

The patient was counseled on avoiding SMX/TMP in the future and was educated on signs and symptoms of hepatotoxicity should he encounter similar reactions with other drugs. Additionally, an alert was placed in his medical record regarding sulfa drug sensitivity. Cross-reactivity with other sulfa-containing medications, although rare, was discussed to ensure a comprehensive understanding of potential future risks [20].

## Conclusions

This case emphasizes the importance of recognizing SMX/TMP as a potential cause of hepatotoxicity, particularly when patients present with jaundice and elevated liver enzymes without alternative explanations. Given the widespread use of SMX/TMP, awareness of its rare but significant hepatotoxic potential is essential for timely diagnosis and intervention. Drug-induced liver injury can mimic other hepatic diseases, so maintaining a high index of suspicion is crucial, especially in cases with recent antibiotic exposure.

Clinicians should consider SMX/TMP hepatotoxicity in differential diagnoses of unexplained jaundice, particularly in high-risk populations, such as the elderly or immunocompromised. Early identification and discontinuation of SMX/TMP, combined with patient education on adverse drug reactions, can prevent severe liver injury and improve patient outcomes. Continued research is needed to better understand the mechanisms behind SMX/TMP-induced hepatotoxicity and identify patient-specific risk factors for this adverse effect.
